# Application of Multimodal Fusion Technology in Image Analysis of Pretreatment Examination of Patients with Spinal Injury

This article has been retracted.

**DOI:** 10.1155/2022/4326638

**Published:** 2022-04-12

**Authors:** Hongliang Wu, Guocheng Chen, Guibao Zhang, Minghua Dai

**Affiliations:** Department of Orthopedics, Pudong New Area Punan Hospital, Shanghai 200125, China

## Abstract

As one of the most common imaging screening techniques for spinal injuries, MRI is of great significance for the pretreatment examination of patients with spinal injuries. With rapid iterative update of imaging technology, imaging techniques such as diffusion weighted magnetic resonance imaging (DWI), dynamic contrast-enhanced magnetic resonance imaging (DCE-MRI), and magnetic resonance spectroscopy are frequently used in the clinical diagnosis of spinal injuries. Multimodal medical image fusion technology can obtain richer lesion information by combining medical images in multiple modalities. Aiming at the two modalities of DCE-MRI and DWI images under MRI images of spinal injuries, by fusing the image data under the two modalities, more abundant lesion information can be obtained to diagnose spinal injuries. The research content includes the following: (1) A registration study based on DCE-MRI and DWI image data. To improve registration accuracy, a registration method is used, and VGG-16 network structure is selected as the basic registration network structure. An iterative VGG-16 network framework is proposed to realize the registration of DWI and DCE-MRI images. The experimental results show that the iterative VGG-16 network structure is more suitable for the registration of DWI and DCE-MRI image data. (2) Based on the fusion research of DCE-MRI and DWI image data. For the registered DCE-MRI and DWI images, this paper uses a fusion method combining feature level and decision level to classify spine images. The simple classifier decision tree, SVM, and KNN were used to predict the damage diagnosis classification of DCE-MRI and DWI images, respectively. By comparing and analyzing the classification results of the experiments, the performance of multimodal image fusion in the auxiliary diagnosis of spinal injuries was evaluated.

## 1. Introduction

Due to continuous development of sensor technology as well as continuous increase of sensor types, the technology of collecting image information and transmitting information through sensors has gradually entered people's field of vision and has become the focus of research. Currently, sensors are used in military and civilian systems. As we all know, different types of sensors transmit different image information, and the collected information is complex and diverse. If multiple types of sensors are used to collect the information of the same image, the information is both complementary and redundant. Information fusion technology is a new science and technology produced by interdisciplinary integration. With the vigorous development of computer technology, the research on information fusion technology has also been further developed [1–4].

Image is the carrier of information, and its fusion plays a key role in many image-oriented technologies, such as concealed weapon detection and product inspection. Image fusion is to combine the information of two or more images into one image according to certain rules. The image eliminates redundant information of the source image as much as possible and contains complementary information so that the information on the image is accurate and complete. The emergence of image fusion technology effectively solves the limitation caused by a single image and enables the information of multiple images to be better utilized. With the rapid development of computer technology, image fusion technology has played a vital role in medical diagnosis, monitoring, transportation, and other fields. Among them, in the research in the medical field, this technology has received extensive attention [5–9].

Medical image fusion integrates image features of different modes and generates new images through certain fusion methods. The new image information is richer and clearer, making up for the defects of a single image. A single medical imaging mode is limited and cannot meet the needs of complex disease diagnosis and treatment. Computed tomography (CT) images mainly reflect high-density tissue information, accurately display the lesion area, and facilitate the determination of the location of the lesion, but its tissue characteristics are very limited. Magnetic resonance imaging (MRI) images have poor image resolution and lack of soft tissue activity information, so they cannot be used as a reference for locating the location of lesions, but they can better present soft tissue imaging information. Positron emission computed tomography (PET) and single-photon emission computed tomography (SPECT) can describe blood flow and significant metabolic changes in the body. However, it lacks organizational and structural information. Obviously, a single-modal medical image can only reflect part of the information of a certain part of the patient, but cannot provide all the information of the part. Usually, doctors need to arrange images of different modalities together in order to get more comprehensive information. According to observation, comparison, and imagination, the information of multiple images is integrated in the brain and then combined with their own experience to judge the patient's condition. This process is prone to errors, and once errors occur, it is likely to cause misdiagnosis to patients [10–14].

Medical image fusion technology fuses images from different sensors and utilizes the complementarity of images from different modalities, which can effectively utilize the imaging characteristics of multiple modalities. The fused image contains various information and can more accurately reflect the structure and function of the patient's body. In this way, doctors can provide more comprehensive and reliable imaging data for diagnosis and follow-up data. Through the information provided, the accuracy of the doctor's diagnosis can be improved. Clinical medicine has confirmed that, through a certain fusion method, the complementary information of multiple single-modality medical images is recombined into one image, which usually produces relatively good results. This work uses machine learning methods to fuse multimodal spine image information for efficient diagnosis of spinal injuries. The key contribution is as follows:

- A registration study using DCE-MRI and DWI image data. To increase registration accuracy, a registration technique is utilized, and the VGG-16 network structure is chosen as the fundamental registration network structure. In addition, an iterative VGG-16 network architecture is presented to accomplish the registration of DWI and DCE-MRI images.
- Based on a study that combined DCE-MRI and DWI image data. This research employs a fusion technique incorporating feature level and decision level to categorize spine pictures from registered DCE-MRI and DWI images. The damage diagnostic categorization of DCE-MRI and DWI images was predicted using the basic classifier decision tree, SVM, and KNN, respectively. The effectiveness of multimodal image fusion in the auxiliary diagnosis of spinal injuries was examined by comparing and evaluating the classification findings of the tests.

## 2. Related Work

The registration algorithms of multimodal medical images can be divided into two categories according to the registration basis. One is the region-based registration method, which is mainly based on the principle of information theory. There is another type of registration algorithm based on image features, which mainly finds the common features of two images based on some feature recognition operators, so as to perform feature alignment registration. Harris features were used to develop a partial intensity-invariant feature descriptor for low-quality picture pairs in [15]. When the UR-SIFT feature was used with the PIIFD descriptor in [16], good results were obtained. Harris-PIIFD may not be able to appropriately align retinal color pictures with other modalities in the face of substantial content changes, according to [17]. For multimodal retinal image registration, SURF-PIIFD-RPM, a robust point matching system, is proposed. The PIIFD descriptor is used to match features extracted from the two pictures using the SURF detector. Once the mapping function is estimated, a single-Gaussian robust point matching model based on the Hilbert space kernel approach is utilized to better match the putative matching set with outliers SIFT and PIIFD outlier suppression techniques were introduced in [18]. A symmetric-SIFT can register CT and MR brain images quickly by stiff transform estimation in addition to the methods listed above [19]. Medical image registration has been revolutionized by the MI technique, according to the literature [20]. If the photos are not properly aligned with each other, the overlap-invariant MI can reach its maximum value. According to [21], a normalized version of MI, NMI, was proposed to better match slices by clinical MR and CT brain imaging volumes. For deformable image registration, the upper bound on the maximum MI has been studied in [22]. This study offers more information about using maximum MI as a similarity metric. CMI is an enhanced, nonrigid registration similarity metric proposed in [23]. Joint histogram of intensity and spatial dimension is based on CMI in three dimensions. To create the histogram, it used a tensor product B-spline nonrigid registration approach in conjunction with the Parzen window and generalized partial volume kernel.

Image fusion means fusing the available information from different sensors into one image. The output of fusion is an image that contains a lot of information, that is, contains a lot of entropy. In [24], a two-scale decomposition image fusion method was proposed, and the base layer and the detail layer were obtained by low-pass filter. Using spatial proximity filters, [25] proposes real-time picture fusion by repeatedly decomposing images into a base and detail layer at various scales. To combine the finer details, researchers in [26] used a multichannel pulse-linked neural network model and a fusion method based on three-scale decomposition. The basis-detail decomposition approach, based on saliency detection, was described in [27] as a fusion strategy. Using alternating directed filtering, a basis-detail decomposition approach was suggested in [28]. In [29], a sparse coefficient fusion technique based on regions was proposed. When a sharpness-enhanced image is created by injecting sharpness information into a normalized version of the source image, the segmented region is used to help fuse sparse coefficients from this image. An image fusion approach based on multicomponent sparse representation was proposed in [30]. The cartoon and texture components of the original image can be represented by analyzing the model using morphological logic components. As a result, it is more adaptable when it comes to developing more effective improvement tactics that take into account the unique properties of various components. An adaptive sparse representation (ASR) model for picture fusion was introduced in [31]. When dealing with noisy images, it is difficult to use a single high-redundant dictionary; therefore, the ASR model instead learns a more compact set of subdictionaries based on different gradient directions. The first time convolutional neural networks were used for image fusion was in [32]. To enhance the network's ability to extract features, a multilevel feature-guided CNN with skip connections was proposed in [33]. Reference [34] proposed the use of spatial domain fusion to combine multiple source images using a pixel CNN model that separated pixels from each source image into three categories: those that were sharply focused, those that were not sharply focused, and those that were unknown. A fully convolutional network-based image fusion approach was proposed in [35]. The full image is used to train the network, resulting in a focus map of the same size as the source image. As a result, a method based on Gaussian filtering is being developed to create supervised learning sources from raw images and focused segmentation maps and treat the fusion task as a segmentation issue.  Table 1 shows the comparison of literature with algorithm used.

## 3. Multimodal MRI Image Registration

The idea of the traditional image registration algorithm is to find the best spatial transformation in which the corresponding points in the physical space of the image and the image are aligned with each other so that the same position points in the corresponding space in different images correspond to each other. For the two images that need to be registered, they are called floating image *A* and reference image *B*, respectively. According to the characteristics of the image, the appropriate spatial transformation function and similarity measurement are selected. After the floating image is spatially transformed, the pixel gray value of each point of the floating image is obtained by using the image interpolation method. By continuously updating the parameters of the spatial transformation *T*, the parameters are optimized to minimize the difference between the floating image and the reference image. The idea of deep learning further expands the traditional image registration methods. Currently, the common deep learning-based image registration methods are mainly divided into two categories. One is to iteratively estimate a similarity measure between two images using a deep learning network. The other is to use a deep learning network to predict the transformation parameters between two images. The former method only uses deep learning to estimate the similarity measure and still uses the traditional registration method in iterative optimization, which does not shorten the registration time. Therefore, this paper adopts the registration idea of the second type of deep learning to register the spine DCE-MRI and DWI images. This work designs an iterative VGG-16 to conduct image registration. In order to introduce the registration method used in this paper more clearly, the following four aspects are introduced: the basic principle of spatial transformation network, the structure of VGG-16 network model, and the iterative VGG-16 network registration framework.

### 3.1. Spatial Transformation Network

Spatial Transform Network (STN) is a new learning model in convolutional neural networks that can be used as a separate module or added anywhere in convolutional neural networks. Since convolutional neural networks cannot truly achieve invariance to large-scale spatial transformations, the spatial transformation network can allow the neural network to actively perform spatial transformation on the features without additional network training so as to realize the invariance of the network model to translation, rotation, and other distortions. The spatial transformation network consists of three parts: localization network, parameterized grid generator, and differential image sampling. The structure of the spatial transformation network is shown in Figure 1.

The input of the spatial transformation network is *U* and the output is *V*. In the local network, the parameter variable *θ* that maps the input image to the output image is obtained, and the relationship between the input image and the corresponding coordinate point of the output image is reflected by *θ*. The grid generation is to generate the coordinate points of the original image according to the parameter variable *θ*:

(1) $$\begin{array}{c} \left(x_{i}^{m}y_{i}^{m}\right)=\Gamma_{\theta }\left(G_{i}\right)=S_{\theta }\left(x_{i}^{n}y_{i}^{n}1\right). \end{array}$$

Among them, *m* represents the coordinate point of the input image, *n* represents the coordinate point of the output image, (*x*_*i*_^*m*^*y*_*i*_^*m*^) is the coordinate of each pixel of the input image, and *S*_*θ*_ is the output result of the local network.

In order to enable the spatial transformation network to back propagate to train the network, the mapping relationship between the output image and the input image is constructed in the resampling, a resampling function that can be reversed gradient calculation is implemented, and the given interpolation method is used to calculate the output image. For the gray value of the corresponding point, the commonly used interpolation method is the bidirectional linear interpolation method.

### 3.2. VGG-16 Model

Although many scholars have studied many convolutional neural network structures to solve the image registration problem, there are few studies on the registration of spine DCE-MRI and DWI modalities. For the registration of a specific image dataset, it is also necessary to select an appropriate network structure to ensure that the network model parameters can be fitted. In order to explore the registration effect of convolutional neural networks on spine DCE-MRI and DWI images, this paper explores the registration effect of DCE-MRI and DWI images based on the VGG-16 network model.

VGGNet is a convolutional neural network constructed for the first time in [36]. VGGNet is an improvement over AlexNet, the model convolution kernel size is 3 × 3, and the number of network layers reaches 16∼19. The 16-layer convolutional neural network is called VGG-16. The 19-layer convolutional neural network is called VGG-19. VGGNet stood out with excellent results in the 2014 ImageNet Challenge, which won the second place in the image classification problem and the first excellent result in the image localization problem. After that, VGGNet is also widely used in various tasks in the image field.

VGGNet is divided into 6 configurations (A ∼ E) according to the number of convolution kernels and convolution layers, where *D* is the VGG-16 network. The VGG-16 structure contains 13 convolutional layers, 1 pooling layer, and 3 fully connected layers. The unit block of the model consists of two or three convolutional layers stacked, ensuring that the size of the data remains the same after the convolution operation. By adding a maximum pooling layer after each block to reduce the size of the input feature map, while retaining the extracted features, the dimensionality of the input data is reduced to reduce the amount of computation in network learning. A fully connected layer with three layers is connected at the end of multiple stacked blocks to obtain all the data features of the previous layer and process classification tasks more accurately. The entire VGG-16 network architecture is shown in Figure 2.

In each unit module block, the convolution kernel size of the convolutional layer is set to 3 × 3, the sliding step size is set to 1, and the peripheral expansion size is set to 1. Before performing the convolution operation, it is necessary to perform the peripheral expansion operation on the input feature map, extract the features in the middle of the feature map multiple times, and dilute the feature extraction around the feature map. By successively stacking multiple convolutional layers in pairs, the features of the image can be better extracted compared to large-dimensional convolutional layers. The ReLU activation function is used for the mapping calculation in each convolutional layer and each final fully connected layer in the VGG-16 neural network. We have inserted Table 2 for tuned parameter.

### 3.3. Iterative VGG-16 Model

Since the data used in this paper do not provide the true value of registration, this paper adopts an unsupervised deep learning registration method to achieve the registration of spine DCE-MRI and DWI images. This section proposes an iterative VGG-16 network model (IVGG16) based on the original VGG-16 neural network model. The entire registration framework is shown in Figure 3, and the registration is mainly divided into two parts. The first part is the first training of VGG-16 for coarse registration. The input of this network is a pair of DCE-MRI and DWI image images. After the pair of DCE-MRI and DWI images to be registered first enters the first layer of the VGG-16 network, the deformation between the DCE-MRI and DWI images is obtained for the first time. According to the deformation field, the DWI image is distorted and deformed to obtain a coarsely registered image. The second part is the second training of the VGG-16 neural network for fine registration. At this time, the input of the VGG-16 network is the coarse registration image and the DCE-MRI image, and the deformation field between the DCE-MRI image and the coarse registration image is obtained again. The warping results in a fine-registered image.

In addition, since the convolutional neural network cannot well realize the invariance of the network model to translation, rotation, and other distortions, the learning of linear transformations such as translation, distortion, and rotation of image morphology is not accurate enough. A spatial transformation network is added after the VGG-16 neural network to guide the image deformation. Finally, to optimize the results of DCE-MRI and DWI image registration, a loss function of mean square error and gradient descent is used. The difference value of DCE-MRI and DWI images is estimated and fed back to the convolutional neural network to realize the registration of DCE-MRI and DWI images.

## 4. Multimodal MRI Image Fusion

To further study the auxiliary ability of spine DWI image and DCE-MRI image fusion in the diagnosis of spine injury, this chapter uses spine DCE-MRI and DWI image fusion as an entry point to study the auxiliary value of spine DWI image information for spine injury diagnosis. In this paper, the image fusion algorithm of feature level and decision level is combined to realize the classification of spine DCE-MRI and DWI image fusion. First, the spine DCE-MRI and DWI image features are fused, and then the learning method in decision level is used to diagnose spinal injuries. By comparing the effects of single-modality image classification, the auxiliary diagnostic ability of fusion DWI images for classification was evaluated.

### 4.1. Single-Modality MRI Image Classification

Support vector machine (SVM) is a linear binary classification algorithm in a broad sense, which can solve linear inseparable classification problems by using kernel functions. As a commonly used algorithm in machine learning, the biggest feature of other classification algorithms is that the classification effect of the SVM algorithm can also achieve good results for data with high-dimensional features. Even when the feature dimension is larger than the number of samples, SVM can maintain good results. The idea of SVM algorithm is to maximize the interval between samples, which is the largest division that can be found on the hyperplane of the sample space.

The problem of finding the maximum value of the sample interval can be transformed into a relatively easy-to-solve convex quadratic programming problem, and the Lagrangian dual problem is introduced to solve the convex quadratic programming problem to determine whether the KKT condition is satisfied. For a given training sample set *D*={(*x*_1_, *y*_1_),…, (*x*_*n*_, *y*_*n*_)}, for such a sample space, the partition of the hyperplane can be defined as

(2) $$\begin{array}{c} w^{T}x+b=0. \end{array}$$

To deal with linearly inseparable classification problems, the features of the samples are usually mapped to a special high-dimensional space. It selects an appropriate kernel function to operate on low-dimensional space so as to avoid complex calculations on high-dimensional space and then solve it.

As one of the classic algorithms in classification algorithms, decision tree algorithm can not only handle regression problems, but also classification problems. The decision tree is based on a tree structure, and the algorithm mainly includes three steps: feature selection, decision tree generation, and decision tree pruning. First, build a decision tree model based on the training set, perform feature selection operation every time the root node and internal nodes are encountered, and select the current optimal division feature for each subdata set. For example, the ID3 algorithm uses information gain as the criterion for feature division. Information entropy is an important indicator to measure the data purity in the sample dataset:

(3) $$\begin{array}{c} E\left(D\right)=-\sum_{k=1}^{\left|y\right|}p_{k}\log_{2}p_{k}. \end{array}$$

Among them, *p*_*k*_ represents the proportion of the *k* class samples in the sample set *D*. When the value of *E*(*D*) is larger, it indicates that the purity of the sample set is higher.

To prevent overfitting during the learning process, the classification ability of the decision tree can be improved by pruning. Start from the root node, select the corresponding output branch according to the feature, end at the leaf node, and finally output the decision result. Although the decision tree algorithm is easy to understand and can get good results in a short time, it is easy to ignore the correlation between each attribute in the dataset.

KNN algorithm is a kind of classification by calculating the distance between different eigenvalues of training data. The idea of the KNN algorithm is as follows: for the input vector that needs to be predicted, find *k* vector sets that are closest to the vector in the training data set, and let input vector be classified as the category with the largest number of categories among these *k* vectors. Euclidean distance is commonly used to calculate the distance between the test set and each training set:

(4) $$\begin{array}{c} \rho =\sqrt{{\left(x_{2}-x_{1}\right)}^{2}+{\left(y_{2}-y_{1}\right)}^{2}}. \end{array}$$

Because there is only one parameter in KNN, the selection of the *k* value directly affects the prediction result, and generally it will not exceed 20. Generally, the *k* value is determined by the cross-validation method. The KNN classification algorithm encounters complex sample sets, which can lead to complex computations.

### 4.2. Fusion Based on Feature Level and Decision Level

Canonical correlation analysis is one of the most common among multivariate statistical methods. So far, extended algorithms based on canonical correlation analysis have been successfully applied to various fields, such as image analysis, data analysis, text mining, classification, and recognition.

Canonical correlation analysis is to find the maximum correlation coefficient between two data. The basic idea of the algorithm is to convert two sets of data into two sets of vectors and use weights to select linear components in the vectors. The correlation coefficient between linear components is calculated by continuously adjusting the weight coefficient, and the linear component with the largest correlation coefficient is found to represent the two sets of vectors. For a given image of DCE-MRI and DWI, modalities are denoted as *D*_1_ and *D*_2_, the training sample space Ω = {*D|D* ∈  *R*^*N*^}, assuming *A* = {*x|x* ∈  *R*^*p*^}, *B* = {*y|y* ∈  *R*^*q*^}, where *x* and *y* are two sets of feature vectors in two different modalities, DCE-MRI and DWI, respectively, and feature fusion is achieved after finding the linear component with the largest correlation coefficient. Suppose *x* and *y* are regarded as random vectors on vector spaces *A* and *B*; first extract the canonical correlation features between *x* and *y*, respectively. The first pair of canonical variables obtained is denoted as *a*_1_^*T*^*x* and *b*_1_^*T*^*y*, and the second pair of canonical variables is denoted as *a*_2_^*T*^*x* and *b*_2_^*T*^*y*. At this point, the requirement of *a*_2_^*T*^*x* and *b*_2_^*T*^*y* is not related to the first pair of *a*_1_^*T*^*x* and *b*_1_^*T*^*y*. Then, *m* regards the typical variables *A* and *B* as transformed feature components:

(5) $$\begin{array}{c} X^{\prime }{\left(a_{1}^{T}x,a_{2}^{T}x,\ldots ,a_{m}^{T}x\right)}^{T}=W_{x}^{T}x,\\ Y^{\prime }={\left(b_{1}^{T}y,b_{2}^{T}y,\ldots ,b_{m}^{T}y\right)}^{T}=W_{y}^{T}y. \end{array}$$

Calculate the cross-variance matrix *C*_*xy*_, covariance matrices *C*_*xx*_ and *C*_*yy*_ of the samples in *A* and *B*, respectively, and the objective function to find the canonical variable with maximum correlation is

(6) $$\begin{array}{c} \underset{a,b}{\max}CCA\left(X,Y\right)=\frac{a^{T}C_{xy}b}{\sqrt{a^{T}C_{xx}ab^{T}C_{yy}b}}. \end{array}$$

To facilitate the solution, a Lagrangian function is introduced to convert the objective function into a convex optimization problem to solve. Take the first *m* pair of projections as typical projection matrices *W*_*x*_ and *W*_*y*_, and finally use the linear transformation matrix to fuse the combined features. Finally, the SVM algorithm is used for classification prediction after fusion of spine DCE-MRI and DWI image features.

Under the premise of image registration, in order to reflect the spinal injury information more comprehensively and accurately, it is necessary to further perform effective fusion processing on the registered DCE-MRI and DWI images. The input and output of the decision-level fusion method are the prediction results of the classifier, which can more effectively obtain real-time classification results. In this paper, three different classification models of decision tree, SVM, and KNN are used to train the registered images, respectively. Retraining is performed according to the prediction results obtained from the initial training, and a fusion algorithm based on the learning method is used to obtain the final classification result.

Due to the different predictive capabilities of different classification models, this paper uses a stacking-based learning method to achieve decision-level fusion. Using three different classification algorithm models, SVM, decision tree, and KNN, as the primary learner of the first layer, all perform the following operations. First, 5-fold cross-validation is performed on each primary learner decision tree, SVM, and KNN, and 4/5 of them are used as the training set and 1/5 as the test set. Each cross-validation is divided into two steps: training the model on the training set and testing the test set according to the model generated by the training. After each cross-validation is completed, keep the training and test data obtained each time as a new training set and test set, which can avoid the phenomenon of overfitting caused by retraining the data. The training data and test data obtained by each classification model are added together and the average is calculated. At this time, a new training set and test set are obtained. The logistic regression algorithm is used as a secondary learner for retraining and testing on the test set to obtain the final classification result, as shown in Figure 4.

In this paper, feature-level and decision-level fusion algorithms are also used to fuse and classify DCE-MRI and DWI images, and the feature fusion images obtained by canonical correlation analysis are used as the input of the stacking learning algorithm. Thus, the fusion classification based on feature level and decision set is realized, as shown in Figure 5.

## 5. Experiment

### 5.1. Evaluation on Image Registration

Due to the different imaging sequences of DCE-MRI and DWI images, the number of image slices is also different. The number of slices in DWI images is generally 34, and the number of slices in DCE-MRI images is generally 190. In order to ensure that each DWI image has a unique DCE-MRI image corresponding to it, it is necessary to screen out the DCE-MRI slice corresponding to the physical location of each patient's DWI slice. Since the filtered image data is less, in order to avoid overfitting during training, it is necessary to use image augmentation technology to generate new data samples on the dataset to expand the total number of samples in the dataset. Commonly used image augmentation methods include flipping, rotating, scaling, cropping, translation, and contrast transformation. To preserve more pixel information on the images, the datasets are augmented with simple flips, rotations, and cropping for DCE-MRI and DWI images, respectively. First, the DCE-MRI and DWI images were flipped horizontally, and secondly, the DCE-MRI and DWI images were rotated by 90° and 180° without changing the image size. Finally, randomly crop the filtered DCE-MRI and DWI images, set the width and height of the cropping frame to 1/4 of the original image, and then enlarge the cropped image to the size of the original image. The final dataset information is illustrated in Table 3.

Because it is difficult to obtain the real deformation field of each test sample data, the transformation parameters of each pixel cannot be accurately measured. Moreover, there is no single gold standard to evaluate the registration effect in the image registration task. Therefore, in this paper, two quantitative analyses, the Dessian similarity coefficient and the mean square error (MSE), are used to evaluate the registration results. This paper uses the Elastix toolkit in ITK to register the data as the benchmark experiment for this experiment to compare the registration results.

To explore the registration effect of convolutional neural network on DCE-MRI and DWI images, this paper compares the registration effect of VoxelMorph and VGG-16 convolutional neural network structure on DCE-MRI and DWI. And use the SimpleElastix toolkit to perform traditional registration methods as a benchmark experiment for comparison, and use Dice coefficient and mean square error to evaluate the registration results of two modalities of spine DCE-MRI and DWI. The experimental results are shown in Table 4.

It can be seen from the data in the table that the three deep learning-based registration results using VoxelMorph, VGG-16, and the network model proposed in this paper are all better than traditional registration. This once again confirms the feasibility of deep learning in the field of image registration. Comparing the registration effects of the three models of VoxelMorph, VGG-16, and IVGG-16, although the registration effect of the VoxelMorph model is better in the registration of spine DCE-MRI and DWI images, however, only looking at the mean square error, the IVGG-16 model has the smallest mean square error value, and the registration effect is better than other models. Moreover, the performance of the IVGG-16 model on Dice is also the closest to the best VoxelMorph.

### 5.2. Evaluation on Image Fusion

To study the auxiliary ability of spine DCE-MRI and DWI image fusion in the diagnosis of spinal injury, this section mainly verifies its classification effect from two aspects: single modality and multimodality. In the first part, the two kinds of spine DCE-MRI and DWI images were used for the diagnosis of spinal injury using a simple classifier, and their classification performance was evaluated respectively. On the basis of the single-modality image classification experiment, the second part compares three methods of spine DCE-MRI and DWI image fusion and evaluates the diagnostic effect of the fusion method on spinal injury from these three aspects.

This section mainly uses three simple classification algorithms, SVM, DT, and KNN, to classify and predict spine DCE-MRI images and DWI images respectively. The classification and prediction of spine DCE-MRI images and spine DWI images were performed by multiple classification algorithms, and the diagnostic performance of DCE-MRI images and DWI images under different classification algorithms in spinal injuries was compared.

Figure 6 lists the diagnostic performance of spine DCE-MRI images under different classification algorithms. And the results of the four evaluation indicators of classification accuracy (ACC), sensitivity (SE), specificity (SP), and area under the ROC curve (AUC) are given in detail.

By observing the damage diagnosis and evaluation results of different classification algorithms on DCE-MRI images, it can be clearly found that the classification effect of the SVM algorithm is better than that of the DT and KNN classification algorithms in terms of accuracy and AUC. Moreover, under the SVM algorithm, the specificity of DCE-MRI image classification is also the highest. The most sensitive is the KNN classification algorithm. However, the accuracy and sensitivity of the decision tree classification algorithm are the lowest among the three classification algorithms.

Figure 7 lists the diagnostic evaluation results of spinal DWI images under different classification algorithms.

For the classification effect of DWI images, the accuracies of SVM classification algorithm and KNN classification algorithm are similar. But the AUC of the SVM algorithm is the best among the three algorithms. However, the KNN algorithm is the best in terms of sensitivity, and the SVM algorithm is the best in terms of specificity. In the experiments on the classification of spine DWI images, it can still be found that the sensitivity of the SVM classification algorithm and the decision tree algorithm is lower, which is similar to the results of spine DCE-MRI images.

This section investigates the classification performance of spinal DCE-MRI and DWI image fusion to explore the ability of fusion to aid in the diagnosis of spinal injuries. The performance of the fusion classification combining feature-level and decision-level is evaluated by comparing the feature-level fusion algorithm with the decision-level fusion algorithm.

Table 5 details the evaluation results of different algorithms for the diagnosis of spinal DCE-MRI and DWI image fusion. Among them, DF represents the use of canonical correlation analysis to achieve feature-based fusion classification. For the DF algorithm, after feature fusion, in order to avoid the influence of the classification algorithm on this experiment, the SVM classification algorithm is used to diagnose the image damage. SF stands for decision-level based fusion using learning methods. DF + SF stands for a fusion that combines feature-level and decision-level.

The accuracy of the SF algorithm is low because some characteristic information of lesions is lost in the decision analysis. However, the performance of the DF algorithm in terms of sensitivity is the best among the three algorithms, which also shows that the feature-level fusion algorithm can accurately predict the lesions on the premise that the sample set is biased towards benign. The DF + SF algorithm outperforms the other two fusion algorithms in all four performance indicators. This also confirms that combining feature-level and decision-level fusion can improve the performance of spine DCE-MRI and DWI image fusion diagnosis.

## 6. Conclusion

With the gradual penetration of computer technology into various branches of the medical field, smart medical care has also become a hot spot of people's attention today. For traditional medical diagnosis, only relying on the doctor's knowledge and experience to judge the patient's condition is too dependent on the doctor's subjectivity, and the speed of reading the images is also limited by the doctor. The development of artificial intelligence has prompted the method of medical diagnosis to gradually shift to computer-based assisted diagnosis. In intelligent medicine, the fusion of multimodal medical images is an inevitable research point. Through proper fusion processing of multimodal medical images, more detailed information of the lesion location can be obtained, and the accuracy of clinical diagnosis and evaluation of medical images can be further improved. Based on deep learning, this paper mainly studies the registration model and fusion algorithm of DCE-MRI and DWI images of spinal injuries. The auxiliary diagnosis ability of DCE-MRI images combined with DWI image information in spinal injuries was evaluated by comparative experiments. The main work of this paper has the following two parts: (1) the registration study of DCE-MRI and DWI images. Based on the VGG-16 network structure, this paper proposes an IVGG-16 unsupervised registration model to achieve registration between DWI and DCE-MRI images. (2) Fusion study of DCE-MRI and DWI images. This paper proposes a fusion algorithm that combines feature level and decision level. The canonical correlation analysis method is used to realize the fusion based on the feature level, and the learning method is used to construct a stacking framework to realize the fusion based on the decision level. The experimental results verify that the fusion of DCE-MRI and DWI images can help improve the diagnostic performance of spinal injuries.

## Figures and Tables

**Figure 1:** The structure of STN.

**Figure 2:** The structure of VGG-16.

**Figure 3:** The structure of registration network.

**Figure 4:** The structure of learning method.

**Figure 5:** Feature-level and decision-level fusion process.

**Figure 6:** Comparison of diagnostic results of DCE-MRI images for spinal injuries.

**Figure 7:** Comparison of diagnostic results of DWI images for spinal injuries.

**Table 1:** Comparison of literature with algorithm used.

Author and reference	Issue	Method	Results
Chen et al. [15]	Multimodal retinal image registration	Harris-PIIFD	168—pair of retinal images, acceptable rate—89.9% and incorrect rate—0.6%
Ghassabi et al. [16]	Fail to register color retinal images	UR-SIFT-PIIFD	120—pair of retinal images, successful rate—90%, RMSE—2.7%
Wang et al. [17]	Multimodal retinal image registration	SURF-PIIFD-RPM	142—pair of retinal images, acceptable rate—91.55%, and RMSE—8.07%
Tang et al. [34]	Distances in front of or behind the focus plane are defocused and blurred	p-CNN	50000 images for training and 10000 images for testing, acceptable rate—95.95%, and RMSE—2.4%
Yang et al. [33]	Multifocus image fusion	MLFCNN	60 million pair for training and 10 sets multifocus images for testing, accuracy rate—99.84%, and training time—5.0 hours
Ours	Imaging screening techniques for spinal injuries	DCE-MRI	29057—training data and 11059—testing data, ACC—86.00%, SE—91.00%, SP–89.00%, and AUC—87.00%

**Table 2:** Tuned parameters for AI algorithm.

AI algorithm	Tuned parameters
DCE-MRI	VGG-16 CNN—13 convolutional layers, 1 pooling layer, 3 FCC layers, kernel size—3, activation function—ReLU

**Table 3:** The details of dataset.

Training data	Test data	Total
29057	11059	40116

**Table 4:** Comparison of registration experimental result.

Method	Dice	MSE
SimpleElastix	0.72	6.25
VoxelMorph	0.86	4.37
VGG-16	0.78	4.57
IVGG-16	0.85	4.21

**Table 5:** Comparison of diagnostic results of DCE-MRI and DWI image fusion.

Fusion	ACC	SE	SP	AUC
DF	0.84	0.90	0.84	0.85
SF	0.81	0.82	0.87	0.86
DF + SF	0.86	0.91	0.89	0.87

## Data Availability

The datasets used during the current study are available from the corresponding author upon reasonable request.
